# Models of Artificial Intelligence-Assisted Diagnosis of Lung Cancer Pathology Based on Deep Learning Algorithms

**DOI:** 10.1155/2022/3972298

**Published:** 2022-03-26

**Authors:** Su Chen

**Affiliations:** The First Affiliated Hospital, Sun Yat-Sen University, Guangzhou 510030, Guangdong, China

## Abstract

In this article, in order to explore the application of a diagnosis system for lung cancer, we use an auxiliary diagnostic system to predict and diagnose the good and evil attributes of chest CT pulmonary nodules. This research improves the new diagnosis method based on the convolutional neural network (CNN) and the recurrent neural network (RNN) and combines the dual effects of the two algorithms to process the classification of benign and malignant nodules. By collecting H-E-stained pathological slices of 652 patients' lung lesions from two hospitals between January 2018 and January 2019, the output results of the improved 3D U-net system and the consistent results of two-person reading were compared. This article analyzes the sensitivity, specificity, positive flammability rate, and negative flammability rate of different lung nodule detection methods. In addition, the artificial intelligence system's and the radiologist's judgment results of benign and malignant pulmonary nodules are used to draw ROC curves for further analysis. The improved model has an accuracy rate of 92.3% for predicting malignant lung nodules and an accuracy rate of 82.8% for benign lung nodules. The new diagnostic method using the convolutional neural network and the recurrent neural network can be very effective for improving the accuracy of predicting lung cancer diagnosis. It can play a very effective role in the disease prediction of lung cancer patients, thereby improving the treatment effect.

## 1. Introduction

In the last decade, the mortality and morbidity of malignant tumors have been increasing, which has led to a very serious situation in cancer prevention and cancer treatment. From the perspective of cancer incidence, lung cancer has the highest incidence among the top ten cancers, and deaths due to lung cancer ranks first among the top ten cancer deaths. After investigation, it is found that the symptoms of lung cancer are not so obvious in the early stage. The patient does not feel any abnormality in the body at the early stage. Only when the body is abnormal, it is diagnosed as lung cancer. The stage of the patient diagnosed with lung cancer is normally intermediate to advanced stage. For patients in the advanced stage, the current medical level of clinical surgery has no effect, so generally, patients in the late stage will give up treatment, and their survival rate is relative. However, for early lung cancer patients, it can be treated by clinical surgery, and there is a very high survival rate.

Research on the diagnosis system for lung cancer based on text and images can provide reference value for clinicians. It can effectively reduce the workload of clinicians to screen early lung cancer patients manually and prevent missed screening due to fatigue and other factors. It can provide effective tools for the early detection and diagnosis and increase the chance of curing lung cancer patients.

Pulmonary sarcoidosis is a multisystem and multiorgan granulomatous disease of unknown etiology, which often invades the lungs, bilateral hilar lymph nodes, eyes, skin, and other organs, and the chest invasion rate is as high as 80%–90%. In recent years, the application of deep learning algorithms in medicine has developed rapidly, and research in this area has also emerged in an endless stream. Zheng S applied MIP images to improve the efficiency of automatic lung nodule detection using the CNN [1]. Meanwhile, Koning H J investigated this issue and obtained relevant data from the registry. Data analysis showed that in high-risk trials, lung cancer mortality was significantly lower in patients screened with volumetric CT than in untested patients [2]. In the research of deep transfer learning, Zhao tested the deep learning model. For the external test set, the transferred model has good generalization ability [3]. Jae-Hong developed a new CNN-based system combining a pretrained deep CNN structure and a self-training network [4]. Wang proposed a new method for breast cancer screening and diagnosis based on the CNN model. This method produced a CNN-based breast cancer CT image detection model and a breast cancer screening model [5]. Artificial intelligence is also used for auxiliary diagnosis of cervical cancer. Zhu used the TBS report artificial intelligence cervical fluid thin layer cytology auxiliary diagnosis system jointly developed by Southern Medical University and Guangzhou Fuqiang Pathology Technology Co. Ltd. to diagnose all clinical specimens [6]. Although artificial intelligence can achieve good results in medical applications, there are still difficulties in application. Reliable deep learning models require additional effort and cost. To this end, Guo Ke proposed a new medical-aided diagnosis model as a service. This will help medical institutions obtain reliable medical aid diagnostic models quickly and efficiently [7]. Although deep learning is increasingly used in medical diagnosis, it is not without its drawbacks. Compared with traditional algorithms, when the amount of data processed is too large, deep learning algorithms are slower than traditional algorithms, and a series of problems are prone to occur in practical applications. Therefore, we urgently need a more stable and processing power algorithm model [8].

The innovations of this article are as follows: (1) This article uses a multitask deep neural network technology based on three-dimensional convolution, and its advantage is that it can assign weights to similar structures. (2) This article uses an improved 3D U-net system and compares it with the original system. The improved sensitivity and specificity changes were investigated, and it was determined that the improved 3D U-net system is more suitable for lung nodule identification. (3) This article also uses an ROC curve to distinguish invasive adenocarcinoma from noninvasive lung cancer and discusses the further application of the artificial intelligence system in lung cancer diagnosis.

## 2. Artificial Intelligence-Assisted Diagnosis of Lung Cancer Pathology

### 2.1. Medical-Related Technologies

In the medical field, lung cancer-related examinations mainly include CT images to detect lung nodules, CT image descriptions for analysis, and test reports to further test some information such as tumor markers. This section mainly introduces the lung nodules, the principle of CT imaging, the source of the examination description, and the related information of the examination report [9].

#### 2.1.1. Lung Nodules

Pulmonary nodule is a disease of the lung tissue, it occurs in the early stage of lung cancer, it is a granulomatous disease, and the cause is unknown [10]. The CT image of the lung nodules is shown in Figure 1.

#### 2.1.2. CT Image

The expansion of CT is computed tomography. Generally speaking, CT in clinical practice uses X-rays as the radiation source to emit X-rays, and the final tomographic image is X-ray CT. What we need to know is that all processes that can create images and use computers to build tomograms can be called CT [11–13].

The absorption of X-rays by objects plays a major role in CT imaging. A specific detector is used to receive the X-rays that pass through this layer; the received X-rays are converted into visible light through a converter and then converted into digital signals by an analog/digital converter, which are then input to a computer for processing [14]. The principle of CT is shown in Figure 2.

#### 2.1.3. Inspection Report

The test report mainly includes sputum cytology, pleural fluid examination, blood routine examination, and tumor marker screening. Cytology examination of sputum and pleural fluid mainly determines whether there are tumor cells in the sputum and pleural fluid. Routine blood tests include determining the count of white blood cells, red blood cells, and platelets, as well as cell acidity and alkalinity [15]. The inspection items are shown in Table 1.

### 2.2. Image-Processing Technology

#### 2.2.1. Image Enhancement: Binarization

The relationship between white and black is divided into several levels according to the logarithmic relationship, which is called the “gray level”. The range is generally from 0 to 255, where white is 255 and black is 0, so black and white images are also called grayscale images, which are widely used in the fields of medicine and image recognition. Image binarization is a necessary step in pre-image processing. It is mainly to set the gray value of the pixels on the image to 0 or 255, which can eliminate a lot of noise interference, and the entire image will show only black and white visual effects [16–18].

(1) Binary thresholding: The gray value is set greater than the threshold to maxval, and the threshold is set to 0 in other cases.
  (1) $$\begin{array}{c} D\left(\text{a},b\right)\left\{\begin{array}{cc} \text{max val,} & S\left(\text{a},b\right)>\text{threshold,}\\ 0, & \text{other wise}. \end{array}\right. \end{array}$$
(2) Anti-binary thresholding: The gray value is set greater than the threshold to 0, and the threshold is set to maxval in other cases.
  (2) $$\begin{array}{c} D\left(\text{a},b\right)\left\{\begin{array}{cc} \text{max val,} & S\left(\text{a},b\right)\leq \text{threshold,}\\ 0, & \text{other wise}. \end{array}\right. \end{array}$$
(3) Threshold of truncation: The threshold to the gray value is set greater than the threshold, and the threshold setting remains unchanged in other cases.
  (3) $$\begin{array}{c} D\left(\text{a},b\right)\left\{\begin{array}{cc} \text{threshold,} & S\left(\text{a},b\right)\leq \text{threshold,}\\ S\left(\text{a},b\right), & \text{other wise}. \end{array}\right. \end{array}$$
(4) Threshold is 0: The gray value greater than the threshold is unchanged, and the gray value of the threshold is set to 0 in other cases.
  (4) $$\begin{array}{c} D\left(\text{a},b\right)\left\{\begin{array}{cc} S\left(\text{a},b\right), & S\left(\text{a},b\right)>\text{threshold},\\ 0, & \text{other wise}. \end{array}\right. \end{array}$$
(5) Dethresholding to 0: The gray value not greater than the threshold is unchanged, and the threshold gray value is set to 0 in other cases.
  (5) $$\begin{array}{c} D\left(\text{a},b\right)\left\{\begin{array}{cc} S\left(\text{a},b\right), & S\left(\text{a},b\right)\leq \text{threshold},\\ 0, & \text{other wise}. \end{array}\right. \end{array}$$

#### 2.2.2. Image Filtering

In simple terms, image filtering is a method of image noise reduction, which is mainly divided into linear noise reduction methods and nonlinear noise reduction methods. Linear noise reduction methods mainly include box, mean, and Gaussian methods [19]. The nonlinear noise reduction method is mainly median filtering. In the mean method in the linear noise reduction method, the mean filter using the neighborhood mean method is very suitable for removing grain noise in the image obtained by scanning. The domain averaging method can effectively suppress the noise, and at the same time, it also causes the blurring phenomenon due to averaging; the blurring degree is proportional to the radius of the neighborhood. The median noise reduction in the nonlinear noise reduction method is a commonly performed using a nonlinear smoothing filter. Its main function is to change the pixel with a large difference in the gray value of the surrounding pixels to a value close to the surrounding pixel value so as to eliminate the isolated noise points, so the median filter is very effective in filtering out the salt and pepper noise of the image.

Image filtering can be calculated by the formula

(6) $$\begin{array}{c} O\left(i,j\right)=\sum_{m,n}I\left(i+m,j+n\right)\cdot K\left(m,n\right). \end{array}$$

(I,j) is the position of the pixel in the picture; (m,n) is the position/coordinates in the convolution kernel, and the coordinates of its center point are (0,0).

K(m,n) is the weight parameter on (m,n) in the convolution kernel.

I(*i* + *m*,*j* + *m*) is the picture pixel value corresponding to K(m,n); o(i,j) is the filtering/convolution result of (i,j) pixels in the picture.

*(1) Box filtering*. Box filtering is the simplest processing, where all pixels have the same weighting factor.

The core is

(7) $$\begin{array}{c} h=\alpha \left[\begin{array}{ccc} 1 & \cdots & 1\\ \vdots & \ddots & \vdots \\ 1 & \cdots & 1 \end{array}\right]\alpha =\left\{\begin{array}{cc} \frac{1}{\mathrm{hsize}.\text{width}*\text{hsize}.\text{height}}, & \text{normalize}=\text{true,}\\ 1, & \text{otherwise}. \end{array}\right. \end{array}$$

However, when normalize is true, it becomes a mean filter.

*(2) Mean filtering*. The mean filtering method is a method that takes the average of the target pixel to achieve the purpose of filtering. For the pixels to be processed, the mean filtering method selects a template. The template is composed of several adjacent pixels.

Its core is

(8) $$\begin{array}{c} \text{kore}=\frac{1}{{\text{kore}}_{\text{width}}\cdot {\text{kore}}_{\text{height}}}\left[\begin{array}{ccc} 1 & \cdots & 1\\ \vdots & \ddots & \vdots \\ 1 & \cdots & 1 \end{array}\right]. \end{array}$$

*(3) Gaussian filtering*. Gaussian filtering is a linear filtering and an important method for smoothing the image. The image processed by Gaussian filtering looks more natural than the image processed by the ordinary template [20, 21].

There are two main functional forms of Gaussian filtering. The first is a one-dimensional Gaussian filtering function:

(9) $$\begin{array}{c} G\left(x\right)=\frac{1}{\sqrt{2\pi }\sigma }e^{-x^{2}/2\sigma^{2}}. \end{array}$$

The second is the two-dimensional Gaussian filter function:

(10) $$\begin{array}{c} G\left(x,y\right)=\frac{1}{2\pi \sigma^{2}}e^{-x^{2}+y^{2}/2\sigma^{2}}. \end{array}$$

#### 2.2.3. Edge Sharpening

Edge sharpening is an image processing filter that enhances the edge contrast of an image or video. Visually, images with clear boundaries are preferred by users. Edge sharpening mainly includes expansion, corrosion, opening operation, and closing operation. The edge contrast of an image or video is enhanced by edge sharpening, and its sharpness or clarity can be significantly improved [22].

### 2.3. Related Technologies of Deep Learning

In real life, deep learning methods are widely used to extract and analyze image semantic features, laying a solid foundation for the research of image classification technology.

#### 2.3.1. The Emergence of Deep Learning

In 2006, the concept of deep learning was first proposed. It is a complex algorithm. After years of development, there are many deep learning frameworks [23]. A restricted Boltzmann machine (RBM) is a generative stochastic artificial neural network that learns probability distribution over its input set. The first-generation neural network perception model is shown in Figure 3.

Further research on the RBM model is one of the core contents of deep learning and has very important significance [24]. The RBM power model is shown in Figure 4.

RBM is an undirected graph probability model, which is based on power. We combine the power function of the input layer vector *x* and the hidden layer vector *h* to define the joint probability distribution as

(11) $$\begin{array}{c} O\left(x,h\right)=\frac{g^{-power\left(x,h\right)}}{f}. \end{array}$$

The normalization constant is *F*=∑_*x*,*h*_g^−*power*(*x*, *h*)^. The marginal probability distribution of the observable input data *x* is

(12) $$\begin{array}{c} O\left(x\right)=\sum_{h}O\left(x,h\right)\\ =\sum_{h}\frac{{\text{g}}^{-power\left(x,h\right)}}{f}. \end{array}$$

Introducing free power changes (12) into

(13) $$\begin{array}{c} O\left(x\right)=\frac{{\text{g}}^{-\text{freePower}\left(x\right)}}{f}. \end{array}$$

*f*=∑_*x*_*g*^−*freePower*(*x*)^ is used in formula (13), that is,

(14) $$\begin{array}{c} \text{freePower}\left(x\right)=-\text{log}\sum_{h}{\text{g}}^{-power\left(x,h\right)}. \end{array}$$

*θ* is introduced to represent the parameters of the model; taking the logarithm of (13) and deriving it result in

(15) $$\begin{array}{c} \frac{\partial \text{log}O\left(x\right)}{\partial \theta }=-\frac{\partial \text{free Power}\left(x\right)}{\partial \theta }+\frac{1}{f}\sum_{\hat{x}}g^{-\text{freePower}\left(\hat{\text{x}}\right)}\frac{\partial \text{free Power}\left(\hat{x}\right)}{\partial \theta }=\\ -\frac{\partial \text{free Power}\left(x\right)}{\partial \theta }+\sum_{\hat{x}}O\left(\hat{x}\right)\frac{\partial \text{free Power}\left(\hat{x}\right)}{\partial \theta }. \end{array}$$

In order to deal with the difficult RBM calculation problem of the partition function, the approximate value of the log-likelihood gradient ∂log*O*(*x*)/∂*θ* is usually used for training. The sample x ∼ O(x) subject is used for data distribution and the free power gradient on the sample $\hat{x}∼O\left(\hat{x}\right)$ subject is used for model distribution to define the model parameter update rule as

(16) $$\begin{array}{c} P_{\hat{O}}\left[\frac{\partial \text{log}O\left(x\right)}{\partial \theta }\right]=-P_{\hat{O}}\left[\frac{\partial \text{free Power}\left(x\right)}{\partial \theta }\right]+P_{O}\left[\frac{\partial \text{free Power}\left(\hat{x}\right)}{\partial \theta }\right]. \end{array}$$

Among them, O is the model probability distribution, $P_{\hat{O}}$ and *P*_*O*_ are the expected values under the corresponding probability distribution, and $\hat{O}$ is the empirical probability distribution of the training data set. The first term of (16) is relatively simple, and it is generally replaced by training sample expectations; the second term contains samples obtained from model O.

#### 2.3.2. Deep Learning Model: Convolutional Neural Network Model

Convolutional neural networks (CNN) are feedforward neural networks, which are a feature extraction and classification method for images [25].  Figure 5 shows a simple convolutional neural network model.

It can be seen from Figure 5 that, unlike the multilayer feedforward sensor, the convolutional neural network limits the network structure by using the local connection of the receiving area.

(1) Before training, the ownership value of the convolutional neural network is initialized with different small random numbers for supervised training. There are two stages to training a folded neural network:
  (a) In the prepropagation stage, samples are taken from the sample set and input *X* to the network, where *E* is the weight of the network and Y is the mapping function. The information is passed on and the corresponding actual output is calculated:
    (17) $$\begin{array}{c} B_{P}=Y_{n}\left(\cdots \left(Y_{2}\right.\left(Y_{1}\left(XE_{1}\right)E_{2}\right)\cdots \right)E_{n}. \end{array}$$
  (b) In the retrospective phase,
    (18) $$\begin{array}{c} E_{P}=\frac{1}{2}\sum_{j}{\left(Y_{pj}-O_{Pj}\right)}^{2}. \end{array}$$
(2) Activation function. The sigmoid function and tanh function are the first nonlinear activation functions used in neural networks.

The sigmoid function not only increases monotonically but its inverse function also increases monotonously. Therefore, the sigmoid function is very suitable to be used as a threshold function of a neural network, and its function value is between 0 and 1.

The analytical formula of the function is

(19) $$\begin{array}{c} \text{sigmoid}\left(x\right)=\frac{1}{1+r^{-x}}. \end{array}$$

The output value of the tanh function can be scaled nonlinearly in the range of (-1, 1), which is convenient for normalizing the model characteristics.

The analytical formula of the function is

(20) $$\begin{array}{c} T\left(x\right)=\frac{{\text{r}}^{x}-r^{-x}}{r^{x}+r^{-x}}. \end{array}$$

#### 2.3.3. Long- and Short-Memory Neural Network

The structure diagram of long short-term memory (LSTM) is shown in Figure 6, and each line represents a vector. The yellow rectangle represents the activation function in this neural network layer. The pink circles represent point-by-point operations between vectors, such as vector multiplication and vector addition. Compared with other models, the LSTM model can handle the semantics of long-distance context better in text. Therefore, the LSTM model has become the current mainstream word segmentation task model.

#### 2.3.4. Deep Learning Algorithm of 3D U-Net Model

The deep learning algorithm used in this experiment is a 3D U-net model. In this model, each green cuboid is a module. Each module has a fixed network structure (Figure 7), including 3D convolution, normalization, an activation function, and a pooling layer.

## 3. Artificial Intelligence-Assisted Diagnosis of Lung *Cancer* Pathology Experiment and Analysis

### 3.1. Basic Characteristics of Research Objects

This study retrospectively collected H-E-stained pathological sections of lung lesions in 652 patients from three tertiary hospitals, mainly Jiangxi Provincial People's Hospital, from January 2018 to January 2019. There were 301 males (accounting for 46.2%) and 351 females (accounting for 53.8%), ranging from 24 to 92 years old, with an average age of (61.8 ± 10.5) years. Among them, 278 (41.2%) had malignant lesions, 396 (58.8%) had benign lesions, and 674 had lung nodules, where 488 had solid nodules, 186 had subsolid nodules, 124 had partial solid nodules, and 62 had ground glass nodules; 8 had tiny nodules with a diameter of less than 5 mm in the lung nodules, 74 had small nodules with a diameter of 5 mm ≤ 10 mm, and 592 had nodules with a diameter >10 mm. Among them, there were 387 nodules between 10 and 20 mm and 205 nodules between 20 and 30 mm. There were 218 nodules in the upper lobe of the left lung, 99 nodules in the lower left lobe, 156 nodules in the upper right lung, 69 nodules in the middle right lung, and 132 nodules in the lower right lung (details are shown in Table 2).

### 3.2. Detection of Lung Nodules

Of the 652 patients included, there were a total of 674 pulmonary nodules. There were 633 cases of 1 target lung nodule and 20 cases of 2 target lung nodules. Among them, the improved 3D U-net network-assisted diagnosis system detected a total of 674 target nodules, with a detection rate of 100.0% (674/674). Radiologists reported a total of 673 target sections, with a detection rate of 99.9% (673/674), as shown in Table 3.

Figure 8 shows the difference between the AI model, pathologists, and pathology gold standard. The gold standard refers to the dispute between two pathologists with more than 5 years of experience in the diagnosis of lung diseases. The chief physician discusses the final result of the decision.

### 3.3. Diagnosis of Benign and Malignant Pulmonary Nodules

#### 3.3.1. Prediction of Benign and Malignant

In principle, the 674 cases in this study were divided into two groups at a ratio of 3 : 1: a training group and a research group, with 506 cases in the training group and 168 cases in the testing group. The training group data are used to train the benign and malignant classification models of lung lesions, and the test group data are used to test the model. After the model is tested and refined, the performance indicators of the final classification model are recorded.

In this study, the prediction results of the 168 lung nodules in the test group based on the model established by the deep learning algorithm are shown in Table 4.

It can be seen that there are a total of 104 malignant lung nodules, and the model successfully predicted that 96 of them are malignant, accounting for 92.3% of the total. Among them, 8 were misdiagnosed, accounting for 7.7%. Among all 64 benign nodules, the model successfully predicted 53 benign nodules, accounting for 82.8%. 11 cases were misdiagnosed, accounting for 17.2%.

#### 3.3.2. Comparison between AI's and Doctor's Reading

The 3D U-net can be moved in all three directions (image height, width, and channels). At each position, element-wise multiplication and addition provide a numerical value. Because the filter slides through a 3D space, the output values are also arranged in 3D space. The improved 3D U-net, the original 3D U-net, and the doctor's sensitivity, specificity, negative likelihood ratio, and positive likelihood ratio for benign and malignant judgments are shown in Table 5. The three sets of data are compared in pairs, and the two artificial intelligence systems have their own advantages and disadvantages in judging the benign and malignant pulmonary nodules. The improved 3D U-net system has high sensitivity, high specificity, and a positive likelihood ratio of the 3D U-net system, and the overall performance of the latter is slightly stronger. The positive likelihood ratios of the three were 1.21, 2.13, and 2.81, among which that of radiologists was the highest, but none of the three had a high diagnostic value for benign and malignant pulmonary nodules.

The flammability ratio is the ratio of the mass of air to fuel in the mixture. It is generally expressed in grams of air consumed per gram of fuel when burned. The two artificial intelligence systems are used to judge the benign and malignant pulmonary nodules, and the radiologist draws the ROC curve (Figure 9). The AUC area of the 3D U-net system was 0.583 [*P* = 0.02 (<0.05)]. The AUC area of the improved 3D U-net system was 0.729 [*P* = 0.02 (<0.05)]. The improved 3D U-net system has certain accuracy in the diagnosis of benign and malignant pulmonary nodules, and its performance is close to that of radiologists. The AUC area of the radiologist group was 0.794 [*P* = 0.01 (<0.05)]. The accuracy of manual image reading for the diagnosis of benign and malignant pulmonary nodules was higher than that of the two artificial intelligence systems, but the overall accuracy was average.

#### 3.3.3. Using ROC Curve to Distinguish Invasive Adenocarcinoma from Noninvasive Lung Cancer

The ROC curve is used for analysis, and the nodule diameter, CT value, and malignant probability are used as the cutting points for the differential diagnosis of invasive adenocarcinoma and noninvasive tissue (preinvasive lesion/microinvasive adenocarcinoma). They are 11.38 mm, −377.2 HU, and 95%; the corresponding areas under the ROC curve are 0.931, 0.887, and 0.876, and the sensitivities are 87.9%, 79.5%, and 81.6%, respectively. The specificities were 87.5%, 91.4%, and 75.7%, and the accuracy was 88.2%, 85.3%, and 80.8%, respectively (Figure 10). CT value is a measurement unit for measuring the density of a local tissue or organ in the human body, usually called Heinz unit; for air, it is −1000, and for dense bone, it is +1000. The cleavage site is a commonly used linking sequence for fusion proteins in genetic engineering expression systems, and the target protein in the fusion protein can be separated from the peptide segments of the nontarget protein by drug treatment.

## 4. Discussion

In this study, the improved 3D U-net network-assisted diagnosis system detected 674 target nodules, with a detection rate of 100.0% (674/674). Radiologists detected 673 target sections, with a detection rate of 99.9% (673/674). What the radiologist missed was a solid pulmonary nodule located in the basal segment of the right lower lobe, with a diameter of 29 mm and an unclear boundary with the surrounding tissues. If the artificial intelligence system wants to accurately screen out lung nodules and judge their nature, it needs to go through lung parenchymal segmentation, lung nodule detection, lung nodule segmentation, and lung nodule diagnosis—a total of 4 steps. The first 3 steps are responsible for screening and segmenting lung nodules, and the fourth step is to distinguish between benign and malignant lung nodules. Any failure in any of the first 3 steps will result in missed or false detection of lung nodules. When artificial intelligence extracts nodules, compared with isolated solid nodules, the extraction of adhesion pleural nodules and adhesion vascular nodules is more difficult. Pulmonary nodules adhere to the pleura, blood vessels, and other tissues, and their CT values are similar to those of surrounding tissues, which brings great interference to the extraction of the nodules.

In this study, the improved 3D U-net system's, the original 3D U-net system's, and the physician's sensitivity in judging benign and malignant lung nodules was 95.51%, 91.83%, and 85.1%, respectively. The specificities were 34.46%, 58.69%, and 70.15%, respectively. The positive likelihood ratios were 1.21, 2.13, and 2.81, respectively. The negative likelihood ratios were 0.20, 0.22, and 0.23, respectively. The positive likelihood ratios of the three are less than 10, which is of low value. Comparing the two artificial intelligence systems, the improved 3D U-net system has higher diagnostic sensitivity and poorer specificity than the 3D U-net system. Both artificial intelligence systems are based on the use scenarios of the 3D-CNN system to screen for lung nodules. It is designed to detect lung nodules; the algorithm is optimized for sensitivity, resulting in low specificity, and the ability to cut lung nodules is stronger. The improved algorithm has changed with respect to the optimization direction, so its performance is different. Comparing the two artificial intelligence systems to radiologists, the sensitivity of judging the nature of pulmonary nodules is higher than that of radiologists. In terms of specificity, radiologists lead.

The AUC areas for judging benign and malignant pulmonary nodules are 0.583 AUC area of the original 3D U-net system and 0.729 AUC area of the improved 3D U-net system. The AUC area of the radiologist group was 0.794. The original 3D U-net system has low accuracy in judging benign and malignant pulmonary nodules. The improved 3D U-net system and radiologists have certain accuracy in judging benign and malignant pulmonary nodules. The use of the CNN helps improve the accuracy of CT volume measurement and nodule differentiation in patients with lung nodules in computer-aided detection. At this stage, artificial intelligence shows good performance in judging benign and malignant pulmonary nodules and has a very promising application prospect.

The intelligent diagnosis system based on the improved 3D U-net network can automatically detect lung nodules through automatic segmentation of lesions, automatic measurement of quantitative and qualitative parameters, judgment of nodule types, automatic analysis of benign and malignant nodules, etc. This experiment detected 674 cases of pathological lung nodules. The results showed that mixed ground glass nodules and pure ground glass nodules were more common in adenocarcinoma and only solid nodules were seen in squamous cell carcinoma. The accuracy of distinguishing and diagnosing invasive adenocarcinoma and noninvasive adenocarcinoma in groups was based on the standard diameter of the nodule, CT value, and “malignant probability,” which were 88.2%, 85.3%, and 80.8%, respectively.

There are many shortcomings in this study: because it is impossible to obtain the pathological results of all nodules, the gold standard for judging the true and false of nodules in this study was confirmed by three senior chest CT diagnostic physicians after reading the pictures. The comparative analysis with the artificial intelligence system is carried out by two intermediate-level doctors, and there may be more human errors. The detection method of pulmonary nodules is closely related to their density, location, and shape. The analysis of the detection efficiency of this study only considers the density of nodules, and the influence of factors such as the location of nodules is not included in the scope of the study; further experimental studies are needed in the future. It is believed that as the deep learning research driven by big data continues to deepen, new signs are constantly being explored, and new algorithms are constantly being developed; the auxiliary diagnosis value of artificial intelligence auxiliary diagnosis systems will definitely achieve satisfactory results.

## 5. Conclusion

This paper improves the convolutional neural network model on the original basis and applies it to the diagnosis of benign and malignant lung nodules to assist in the diagnosis of lung cancer. In experiments on a large number of samples, it is verified that the improved model used in this study reduces the complexity of the algorithm while increasing the overall lung nodule detection rate and reducing the misdiagnosis rate. It proves that the artificial intelligence-assisted diagnosis system can help clinicians screen and diagnose patients, improve work efficiency, and reduce workload. In this study, a 3D U-net model obtained by fusion of the convolutional neural network (CNN) and the long short-term memory (LSTM) recurrent neural network (RNN) was used. Compared with the single-modal learning method that scholars of comparative research only use CT images, this method can enable the network model to learn more subtle features. The accuracy of this model for predicting malignant pulmonary nodules can reach 92.3%, and the accuracy of predicting benign pulmonary nodules can reach 82.8%, which prove that the system is feasible and effective. Based on the prediction model designed in this paper, it can play a very important role in the diagnosis of lung cancer, and it can also indirectly improve the treatment of lung cancer in the future.

## Figures and Tables

**Figure 1:** CT image of lung nodules.

**Figure 2:** CT principle.

**Figure 3:** The first-generation neural network perception model.

**Figure 4:** RBM power model.

**Figure 5:** Convolutional neural network.

**Figure 6:** LSTM network structure diagram.

**Figure 7:** Improved 3D U-net model diagram.

**Figure 8:** Pathological gold standard, AI model, and pathological regions segmented by pathologists (black line: AI model, gray line: gold standard, and white line: pathologist).

**Figure 9:** ROC curve of artificial intelligence reading and physician reading.

**Figure 10:** ROC curve of diameter, CT value, and malignant probability.

**Table 1:** Inspection items.

	Reference range	Inspection name	State	Result value
Blood routine examination Sputum examination	0–0.10	Basophils	Normal	0.02
	0.05–0.5	Eosinophils	Normal	0.06
	0–1	Basophil ratio	Normal	0.30%
	110–160	Hemoglobin	Normal	135 g/L
	100–300	Platelets	Normal	158 g/L
	3.5–5.5	Red blood cells	Normal	3.94
	37–50	Erythrocyte distribution width	Normal	45.31%
	4–10	White blood cells	Normal	7.21 g/L
	86–100	Mean red blood cell volume	Normal	89.4 fL
	No tumor cells	Sputum cells	Normal	No tumor cells

Tumor markers	<5 g/ml	CEA	Normal	2.36 g/ml
	<30 U/ml	CA125	Normal	12.5 U/ml
	<8.20 U/ml	CA72-4	Normal	2.24 U/ml
	<16.3 ng/ml	NSE	Normal	14.15 ng/ml
	<1.5 ng/ml	SCC	Normal	1.17 ng/ml
	<2.0 ng/ml	CYFRA21-1	High	6.38 ng/ml

Hydrothorax examination	0.38–2.1	Triglyceride	Normal	0.68 mmol/L
	0.8–1.95	High-density lipoprotein	Normal	1.23 mmol/L
	3.8–6.1	Glucose	High	10.08 mmol/L
	2–4	Low-density lipoprotein	Normal	1.76 mmol/L
	109–271	Lactate dehydrogenase	Normal	174.1 U/L
	0–6.8	Direct bilirubin	Normal	3.18 umol/L
	3.6–5.9	Total cholesterol	Low	3.36 mmol/L
	20–45	Globulin	Normal	33.5 g/L

**Table 2:** Basic characteristics of lung nodules.

Features	Classification	Number of nodules	Proportion (%)
Density classification	Reality	488	72.4
	Partial realness	124	18.4
	Ground glass	62	9.2

Position	Upper lobe of left lung	218	32.3
	Lower lobe of left lung	99	14.7
	Upper lobe of right lung	156	23.1
	Middle lobe of right lung	69	10.2
	Lower lobe of right lung	132	19.6

Diameter	*d* < 5 mm	8	1.2
	5mm d ≦ 10 mm	74	11.0
	10 mm d ≦ 30 mm	592	87.8

Pathological type	Benign	396	58.8
	Malignant	278	41.2

Gender	Male	301	46.2
	Female	351	53.8

Age	Age 24–92 years old; average age (61.8 ± 10.5) years		

**Table 3:** Pathological types of lung nodules.

Pathological types of pulmonary nodules	Number of nodules	Proportion (%)
Benign nodule	396	58.8
Tuberculoma	313	46.4
Hamartoma	62	9.2
Sclerosing alveolar cell tumor	21	3.1
Malignant nodule	278	41.2
Adenocarcinoma	259	38.4
Squamous cell carcinoma	19	2.8
Total	674	100.0

**Table 4:** The prediction results of 168 benign and malignant lung nodules by the deep learning algorithm model.

Pathology	Forecast		Total
	Malignant	Benign	
Malignant	96 (TP)	8 (FN)	104 (P)
Benign	11 (FP)	53 (TN)	64 (N)
Total	107	61	168

Note: TP : true positive. FN : false negative. TN : true negative.

**Table 5:** Comparison of benign and malignant judgments between the improved 3D U-net, the original 3D U-net, and the physician.

Object	Sensitivity	Specificity	Positive fuel-like ratio	Negative fuel-like ratio
Improved 3D U-net	95.51%97.22–95.46%	34.46%27.86–46.85%	1.211.05–1.39	0.200.10–0.35
3D U-net	91.83%82.70–92.37%	58.69%47.33–66.95%	2.131.47–2.48	0.220.10–0.35
Physician	85.1%76.43–88.67%	70.15%60.22–75.68%	2.812.16–3.64	0.230.10–0.35

## Data Availability

No data were used to support this study.
